The article "Greenhouse Gas Emission: Perception during the COVID-19 Pandemic" was published in 2022. Journal: Biomed Res Int.

# Greenhouse Gas Emission: Perception during the COVID-19 Pandemic

**DOI:** 10.1155/2022/6166276

**Published:** 2022-09-30

**Authors:** Kingsley Eghonghon Ukhurebor, Uyiosa Osagie Aigbe, Robert Birundu Onyancha, Gladys UK-Eghonghon, Vincent Aizebeoje Balogun, Peter Eshioke Egielewa, Blessed Frederick Ngonso, Otolorin Adelaja Osibote, Simon Ejokema Imoisi, Juliana Ngozi Ndunagu, Heri Septya Kusuma, Handoko Darmokoesoemo

**Affiliations:** ^1^Department of Physics, Faculty of Science, Edo State University Uzairue, P.M.B. 04, Auchi, 312101 Edo State, Nigeria; ^2^Department of Mathematics and Physics, Faculty of Applied Sciences, Cape Peninsula University of Technology, P.O. Box 1906, Cape Town, South Africa; ^3^Department of Technical and Applied Physics, School of Physics and Earth Sciences Technology, Technical University of Kenya, P.O. Box 52428-00200, Nairobi, Kenya; ^4^Department of Nursing Services, University of Benin Teaching Hospital, P.M.B., 1111 Benin City, Nigeria; ^5^Department of Mechanical Engineering, Faculty of Engineering, Edo State University Uzairue, P.M.B. 04, Auchi, 312101 Edo State, Nigeria; ^6^Department of Mass Communication, Edo State University Uzairue, P.M.B. 04 Auchi, 312101 Edo State, Nigeria; ^7^Department of Public and International Law, Faculty of Law, Edo State University Uzairue, P.M.B. 04, Auchi, 312101 Edo State, Nigeria; ^8^Faculty of Sciences/Africa Centre of Excellence on Technology Enhanced Learning (ACETEL), National Open University of Nigeria, Abuja, Nigeria; ^9^Department of Chemical Engineering, Faculty of Industrial Technology, Universitas Pembangunan Nasional “Veteran” Yogyakarta, Indonesia; ^10^Department of Chemistry, Faculty of Science and Technology, Airlangga University, Mulyorejo, Surabaya 60115, Indonesia

## Abstract

The period 2020/2021 was an unprecedented and historic time for industrial, economic, and societal activities all over the world with great challenges to human health, the ecosystems, and other aspects of human endeavors owing to the COVID-19 or SARS-CoV-2 (CV-19) pandemic which is now a topical aspect of research interest. Despite the negative impacts of the CV-19 pandemic, there are also positive reports during the CV-19 pandemic such as the reduction of gas flare, reduction in the burning of fossil fuels from automobile exhaust and a reduction in the other ensuing factors of greenhouse gases emissions (which is one of the major drives for global warming and climate change as well as other environmental effluences). Hence, this brief perspective review study is centered on greenhouse gas (GHG) emission. The study employs a methodical approach to analyze some already available research studies from existing publications and databases on GHG emission using the perception during the CV-19 pandemic. The specific findings from this review show that, from the meteorological perspective, the global response to the catastrophe ensuing from the CV-19 pandemic has a great influence on the reduction of GHGs, the reduction in the burning of fossil fuels from automobiles and industrial devices, and the reduction in the other ensuing factors of GHG emission. Hence, it will not be far from the truth to conclude that there is a possible positive connection between the CV-19 pandemic and GHG emissions. The study has a direct impact on the environment owing to the negative and positive environmental consequences of the CV-19 pandemic. Suggestions and recommendations in the form of future prospects of GHG emission vis-à-vis global warming and climate change are also discussed. Furthermore, suggestions on how to improve food security and agriculture during a pandemic such as the CV-19 outbreak period are highlighted.

## 1. Introduction

The COVID-19 also known as SARS-CoV-2 (CV-19) which is the short form of the “Severe Acute Respiratory Syndrome Coronavirus-2” is a category of infectious/communicable virus (disease), characteristically instigated by the CV-19 virus which was first discovered and reported at the end of the last month of 2019 in one of the commercial cities of China (Wuhan to be specific). Owing to the deadly and rapidly spread nature of the CV-19, the “World Health Organization (WHO)” declared it a global pandemic on 11 March 2020 [1, 2].

Globally, the CV-19 pandemic caused unprecedented consequences to industrial, economic, and societal activities with great challenges to human health, the environment, agriculture as well as food security, and other endeavors [3, 4]. In addition to the pandemic's debut in 2020, numerous countries experienced food insecurity as a result of financial hardship and rising food prices. Most developing countries have been impacted by macroeconomic issues such as rising inflation and currency exchange rates. Due to the growth in production costs in recent years and during the epidemic, the per capita income of the majority of developing nations was dramatically reduced, and growing inflation and the dollar exchange rate raised the prices of different foods and beverages [5]. Food security was immediately put at risk by food shortages and related price increases, and it was also put at risk by oversupply, which resulted in lower prices for some products and financial losses for farmers and producers [6–8]. According to a report from the “Food and Agriculture Organization of the United Nations (FAO)” during the genesis of the CV-19 era, although the full effects of CV-19 and the novel coronavirus that causes it on agricultural food systems and food security are not yet known, it is obvious that this outbreak will have serious adverse effects on people everywhere along the food supply chain [9]. The import-export restrictions created obstacles for the movement of food, and consumers and producers struggled as a result, which ultimately resulted in a decline in farmer revenue and significant harm to agriculture [9]. However, environmental restrictions like climate change and water scarcity present a challenge to the agricultural sector [6, 10].

Reportedly, the developed regions of the world such as countries in America and Europe were the ones that were mostly, severely, and critically affected during the peak of the CV-19 pandemic, that is, between March 2020 and July 2020 compared to most of the developing regions such as countries in Africa [2]. Even since, there have been several established and reported measures on mitigating the risks associated with the CV-19 as well as other deadly diseases [11]. At the moment, various vaccines have also been discovered, but from all these, it is still alleged that to completely eliminate this deadly disease (CV-19) would take some years. Hence, CV-19 is an issue that the world would conceivably be confronted with for the impending years to come [3, 12, 13].

Despite the several adverse impacts of CV-19 on the environment such as the global increase in the generation of harmful and infectious biomedical waste through the use of personal protective equipment (PPE) and other tools [14–16], the global rise in the manufacture, use and random disposal of safety devices [17, 18], the increase in the generation of municipal/metropolitan solid waste [2, 19], the reduction of recycling of waste [2, 16], and environmental effects and impacts of CV-19 include the massive amounts of sanitizers (disinfectants) that are being used worldwide to eradicate CV-19. An imbalance in the environment could result from the extensive use of these disinfectants, which could lead to the extinction of some useful species that are not targeted [4, 15]. However, several measures to properly dispose of biomedical waste, especially the hazardous and infectious ones generated during CV-19, have been identified in some existing studies [20–22]. There are also reports on the positive impacts of CV-19 on the environment such as the diminution in air pollution and release of greenhouse gases (GHG) [16, 23, 24], diminution in water pollution [25], diminution of noise pollution [2], ecological restoration, and modification of tourist sites [2, 19].  Figure 1 summarizes both the positive and negative environmental effects of CV-19 [26].

As summarized from existing publications by Ukhurebor et al. [4], some of the reported key quantitative issues of the CV-19 virus, especially as they relate to environmental issues, are as follows:

- Given that society resilience depends on an ecological support system with a strong resilience, the CV-19 pandemic emphasizes the connections between natural and societal organizations even more
- The intensification of the food system and the loss of biodiversity are contributing to the rise of zoonotic illnesses
- Environmental factors including air quality appear to have an impact on the effects of the CV-19 virus and are frequently tied to social disparities
- Unwanted effects include increased reliance on plastics alone and a decrease in gasoline prices as a result of lockdowns
- Even though these effects are anticipated to be brief, the lockdowns during the CV-19 pandemic may have some immediate, brief positive effects on the environment, particularly in terms of GHG emission and the quality of the air

However, it is proposed and advised that an additional study is required in order to link the detected evidence and reported environmental changes to the CV-19 virus [27]. Nevertheless, this facile but brief review study will be centered mainly on the gas flare (GF), burning of fossil fuels (BFFs) from automobile exhaust, and other industrial activities as well as other ensuing factors responsible for GHG emission during the CV-19 pandemic. Reportedly, there was a drastic reduction of GHG emission during the CV-19 pandemic [4, 24]. Undoubtedly, GHG emission is one of the major drives for global warming (GW) and climate change as well as some other environmental effluences presently been faced by humanity [28–30]. Consequently, there is a need to constantly develop innovative approaches in mitigating these ensuing environmental effluences resulting mostly from human activities such as GF, the BFFs from automobile exhaust, and other industrial activities as well as the other ensuing factors responsible for GHG emission. One of such ways of developing innovative approaches is to review existing reports/publications and improved on them accordingly. Therefore, this facile but brief perspective review study is centered on GF, the BFFs from automobile exhaust, and the other ensuing factors responsible for GHGs emission drawn from existing publications using the viewpoint during the CV-19 pandemic. Momentarily, the way forward in terms of future prospects in the form of suggestions and recommendations on measures for the mitigation and reduction of GF, the BFFs from automobile exhaust, and the other ensuing factors responsible for GHG emission vis-à-vis GW and climate change has also been discussed.

### 1.1. The Aim, Objectives, and Environmental Significance Statement of the Study

This review study is centered on most of the ensuing factors responsible for GHG emission, drawn from existing publications using the viewpoint during the CV-19 pandemic. The study employs a methodical approach to analyze some already available research studies from existing publications and databases on GHG emission using the perception during the CV-19 pandemic. The study has a direct impact on the environment owing to the negative and positive environmental consequences of the CV-19 pandemic. Allegedly, these positive atmospheric environmental consequences are momentary. However, from all the reports on the influence of CV-19 on the environment, it will not be far from the truth to conclude that there is a possible positive connection between the CV-19 pandemic and GHG emission. The pertinent question is that, *since the* CV-19 *pandemic era experienced some level of environmental boost, should we now crave for the pandemic to continue?* Of course not. From the authors' respective personal viewpoints, all we have to do to sustain these environmental boosts relished during the CV-19 pandemic era is the *green economy*. Consequently, to protect the environment, the combined effort of the countries should be domineering. It is therefore suggested that further advanced studies that would evolve the conduct of nanotechnological (NanoTech) and nanobiotechnological (NanoBTech) research to extenuate the impacts of global warming regarding climate change and other environmental complications should be carried out. The positive influence of the CV-19 pandemic on the environment should be strengthened, to align and capitalize on the ensuing positive consequences of CV-19 for future prospects. Suggestions and recommendations in the form of future prospects of GHGs emission vis-à-vis GW and climate change are also discussed. Furthermore, suggestions on how to improve food security and agriculture during a pandemic such as the CV-19 outbreak period are highlighted.

## 2. GHG Emission: Effects and Possible Relationship with GW and Climate Change

GHGs are gases that trap atmospheric heat. They are gases that possess the ability to absorb or engross infrared radiation (that is, the net thermal energy) emitted or released from the surface of the earth and reradiating it back to the surface of the earth, consequently instigating and contributing to what is known as the greenhouse effect [31]. The furthermost critical GHGs are carbon dioxide (CO_2_), methane (CH_4_), and water vapor. While to a small degree, surface-level ozone (O_3_), nitrogen oxides, and fluorinated gases (especially the chlorofluorocarbons (CFCs), hydrochlorofluorocarbons (HCFC), and halon as well as synthesized sulphur hexafluoride (SHF), hydrofluorocarbons (HFC), nitrogen trifluoride, and perfluorocarbons) also can trap infrared radiation [31].

GHGs have a reflective influence on the energy budget of the earth's arrangement despite comprising only a segment of all gases in the atmosphere. The concentrations of GHGs have changed considerably all through the history of the earth, and these modifications have driven considerable changes in the earth's climate system. Generally, concentrations of GHGs have been predominantly high throughout the warm eras and low (minor) throughout the cold eras. Several processes influence the concentrations of GHGs. Some, like the tectonic actions, run at millions of years, while others, like soil, vegetation, wetland, and water sources as well as sinks, run at hundreds to thousands of years. Since the revolution of industries, human actions, particularly GF and the combustion of fossil fuel are mostly accountable for the steady rise in the concentrations of atmospheric GHGs, specifically CO_2_, CH_4_, O_3_, and the CFCs. The influence of each of the GHGs on the climate system of the earth depends on their chemical nature as well as their relative atmospheric concentration [32–34].

Some of these GHGs have a very high capacity for engrossing infrared radiation or ensue in substantial amounts, while others have substantially lesser capacities for absorption or ensue only in trace quantities. As defined by the “Intergovernmental Panel on Climate Change (IPCC),” radiative forcing is a measure of the effect a certain GHG or other climatic influence (like albedo or solar irradiance) has on the quantity of radiant or solar energy striking, impinging, or interrupting upon the surface of the earth. For a proper understanding of the relative effect of each of the GHGs, the supposed values of the radiative forcing that is measured in watts per square meter (W/m^2^) should be calculated and considered [32].

Shown in Table 1 is the emission sources of some of the utmost GHGs as summarized from some publications [28, 31–36]. Each GHGs' effect on climate change depends on the three foremost factors [31]:

- The amount in the atmosphere: the concentration, or abundance of GHG, is the quantity of the particular GHG in the atmosphere or air. A higher amount of the emissions of GHGs lead to more concentrations in the atmosphere. GHG concentrations are measured in parts per million (ppm), parts per billion (ppb), and even parts per trillion (ppt). 1 ppm is equal to a drop of diluted water into approximately 13 gallons of fluid
- The duration of their stay in the atmosphere: each of these GHGs can stay in the air for different lengths of time, say between a few years and several of hundreds of years. All of these GHGs can stay in the atmosphere for a long duration and become well mixed, implying that the quantity that is measured in the atmosphere is approximately the same globally, irrespective of the cause of the emissions
- The magnitude of their impact on the atmosphere: some of these GHGs are more active than the others in making the earth hotter and in what is known as the “thickening the earth's blanket”

For each GHG, what is known as the “Global Warming Potential (GWP)” is always been calculated to replicate the average duration it stays in the atmosphere and how powerfully it engrosses solar energy. GHGs with a higher GWP engross more solar energy, per pound, than the ones with a lesser GWP, and consequently contributing more to the earth's warming known as GW [31].

## 3. The Impacts of CV-19 on the Environment: Quantitative Perceptive

According to reports, the CV-19 pandemic had a devastating impact on human health and the various mechanisms of the ecosystem (water, soil, and air) as shown in Figure 2 [26].

Globally, as of March 2021, there were approximately 1.17 × 10^6^ persons that were reported and confirmed to have been affected by the CV-19 virus, and the number of related death cases was reported to be around 2.60 × 10^6^ [4]. Since the time that the *WHO* declared CV-19 a global pandemic (that is, 11 March 2020), there have been several reported publications on the environmental impacts of CV-19 globally. Shown in Figure 3 is the various publications in indexed journals as retrieved from the Scopus database using the short statement “environmental impacts of CV-19” over the last year (from 2020 to 12 October, 2021).

The CV-19 virus altered the approach of living as well as the work-related issues for both individuals and the environment, as the various health and managing approaches in securing the restrictions kept several persons indoors. These far-reaching modifications in human activities caused several environmental consequences, as described through the evaluations of the “remote sensing data (RSD)” previously and during the CV-19 pandemic era retrieved from the various environmental agencies and establishments such as “the American Geophysical Union (AGU), the United States Geological Survey (USGS), the National Oceanic and Atmospheric Administration (NOAA) of the US, the European Space Agency (ESA), the National Aeronautics and Space Administration (NASA), the Earth-observing satellites (EOS), and the West African Science Service Center on Climate Change and Adapted Land Use (WASCAL).” As accounted in several reported publications on the environmental impacts of CV-19, there was a rapid modification in environment settings, and the control of this modification seems to indicate that the CV-19 pandemic was conceivably one of the foremost reasons. The degrees of desertification were altered, and the rate of air and other environmental pollutions were suggestively reduced. Consequently, the quality of air and water was improved during the CV-19 pandemic in several regions. However, it was reported by the *WHO* that there is hardly any convincing evidence of a direct relationship between the source, initiation, or transmission of CV-19 virus and GW vis-à-vis climate change, as practically all prevailing pandemics was initiated naturally (especially through wildlife) and facts to indications that human activities could partly drive the initiation and transmission of most of the deadly diseases [4, 23, 26, 37–40]. Globally, the transmission of the CV-19 virus has continued in all regions (cold, temperate, and dry) in respect of the climatic conditions (humid, tropical, and warm climate). Supposedly, the CV-19 virus is principally transmitted from person to person through close interaction or through the respiratory droplets that are formed from infected persons. Also, one can be infected by touching the surfaces which were exposed or affected by the CV-19 virus. Albeit, some weather variables like temperature, pressure, and humidity can conceivably influence the extent of existence of the CV-19 virus outside of the human body, although the influence of weather variables in this regard is anticipated to be trivial when compared to the degree of interaction amongst persons [4, 40–42]. Therefore, it will be more positive to declare that GW vis-à-vis climate change circuitously affected the responses to the CV-19 pandemic by the dejection of the environmental issues of health and the engaged additional pressure on the health arrangements.

Air pollution is one of the causes of most of the critical health threats confronting human health [38]. According to reports air pollutions are mostly instigated through the burning of fossil fuels, GF, and the operation of petroleum-related products, which is one of the foremost drives of GW vis-à-vis climate change. The pollution in the air accounts for the death of around 7.00 × 10^6^ persons every year and is primarily accountable for approximately 34.00% of all deaths from stroke, lung cancers, and all other critical heart diseases [2, 43].

The efforts that were undertaken for the mitigation of the spread of the CV-19 virus reduced most commercial activities, resulting in momentary enhancements in the quality of air in some places, particularly towns and cities. The amount of CO_2_, as well as other GHGs, observed in most of the observation stations in the initial period of the year 2020 was reported to be more than that of the period of the same year, where the CV-19 pandemic was at its peak [26]. Expectedly, the CV-19 pandemic posed enduring adverse environmental effects in the future to come. The excessive use of chemicals substances (like soaps, detergents, and disinfectants), medical drugs, and plastic material substances (like PPE, gloves, facemasks, and syringes) led to a rise in environmental effluences.

Summarily, as adopted and modified from [4], the following are some of the reported critical quantitative perceptive of the CV-19 virus, particularly the ones that relates to its impacts on the environment regarding GW and climate change drawn from the reviewed existing publications:

- The CV-19 pandemic further highlights the interrelations amongst the societal and natural systems. Subsequently, societal resilience depends on a robust environmental support association
- Regular and consistent interconnected to social modifications, environmental structures such as the quality of the air appear to affect the consequences of the CV-19 virus
- Biodiversity loss and the rigorous food establishments make zoonotic viruses more possible
- The rise on the dependency solely on usual of plastics and the drop in the prices of petroleum resource during the CV-19 pandemic have several negative consequences
- The CV-19 pandemic period conceivably has some direct, momentary, and beneficial environmental influences, specifically the reduction in GHG emission in addition to the momentary improved air quality

## 4. GHG Emission during the CV-19 Pandemic

During the CV-19 pandemic, transportation and most industrial activities were halted, and this brought an unanticipated reduction in GHG emission when compared to the pre-CV-19 period. The amount of global air pollution especially in developed regions was relatively reduced by about 50.00% owing to the procedures that were put in place for controlling and managing the dreaded CV-19 virus [16, 23, 24, 44, 45]. As reported by the “United States Environmental Protection Agency (USEPA)” about 80.00% of the GHGs emission such as NO_2_ is instigated as a result of the burning of fossil fuels from automobile exhaust. These GHGs that are emitted (particularly NO_2_) are typically responsible for most respiratory infections and are also accountable for the acid rain interfering with air water and oxygen gas [46]. In an assertion of this, the “European Environmental Agency (EEA)” reported that owing to the decrease in the transportation and most industrial activities the peak of the CV-19 pandemic, NO_2_ emissions dropped from about 60.00% to around 30.00% in most cities in Europe such as Barcelona, Belgrade, Berlin, Brussels, Bucharest, Budapest, Birmingham, Cologne, Hamburg, Istanbul, Kharkiv, London, Madrid, Milan, Minsk, Moscow, Paris, Prague, Rome, Saint Petersburg, Sofia, Tbilisi, Vienna, and Warsaw [47]. According to Berman and Edisu [48], during the peak of the CV-19 pandemic, there was a comparative decline of around 25.50% in NO_2_ emissions in the US compared to the previous era. Similarly, [49] reported the decrease in the degree of NO_2_ in Ontario (Canada) from approximately 4.50 ppb to about 1.00 ppb during the peak of the CV-19 pandemic compared to the previous era. Also, [50] reported that around a 54.30% drop of NO_2_ was noticed in Sao Paulo (Brazil) during the peak of the CV-19 pandemic compared to the previous era. Similarly, during the peak of the CV-19, there was a reported decrease in the amounts of particulate matter 2.5 and NO_2_ by approximately 70.00% in Delhi (India) [51].

Evidently, automobiles and aeronautics are the greatest contributors to GHG emission; they account for about 72.00% and 11.00%, respectively, of GHG emission in the transport sector [45]. Also, the global measure of aeronautical decrease taken for the management and control of the CV-19 had a dramatic influence on the aeronautics sector, since most countries restricted international travelers from entering and exiting in their respective countries, and this helped in the drop in the global CO_2_ emissions of which had critical consequences on the ecosystem especially the atmospheric settings [52, 53]. Supposedly, the significantly less utilization and use of fossil fuels decrease GHG emission, and this eventually assists in the extenuation of global discrepancies in atmospheric settings (climate change) [28, 54, 55]. The “International Energy Agency (IEA)” reported that the global quest for petroleum resources dropped comparatively to around 4.35 × 10^5^ barrels in some months in 2020, when compared to similar months in 2019 [47]. Similarly, the worldwide utilization of coal (apparently, the worldwide coal-based power generation in several nations like China which is one of the main users of coal) was reduced considerably during the CV-19 pandemic owing to the reduction in the demand for energy [44]. Furthermore, Carbon Brief (a British-based meteorological and policy website) reported that owing to the CV-19 issues, there was a reduction in the emissions of CO_2_ in China. The report also anticipates that during the CV-19 pandemic the global amount of CO_2_ was reduced by 4.00% compared to that of 2019 [56].

Also, the recent gas flare data from the “World Bank's 2020 Global Gas Flaring Tracker” from the raw data that was retrieved from 2 satellites managed by the NOAA show a drastic reduction in the gas flared during the CV-19 pandemic era (that in 2020); it was observed that there was a decline in the production rate of petroleum resource by 8.00% (from 8.20 × 10^7^ barrels per day in the year 2019 to 7.60 × 10^7^ barrels per day in the year 2020), with a corresponding decrease in gas flaring by 5.00% between 2019 and 2020 (from 1.50 × 10^2^ bcm in the year 2019 to 1.42 × 10^7^ bcm in the year 2020) (see Figures 4 and 5) [57].

Any of the reported short-term environmental benefits resulting from the CV-19 virus come at an undesirable human and economic rate, and there is hardly any substitute for strategic and sustained action on the quality of air and the climate. Even though some encouraging impacts of the CV-19 virus on the environment were reported, the interim effects were brought by the worldwide lockdown. The environmental boosts resulting from the response to the CV-19 pandemic have now be reversed as the swift increase in economic activities began to come. As suggested by [27, 40], if we are to sustain these environmental boosts relished during the CV-19 pandemic era, there should be a clear prominence that will promote fairness, sustainable environmental safety based on a just evolution in what identified as “green economy.”

## 5. Possible Link between GHG Emission and Food Security and Agriculture during CV-19

The CV-19 pandemic is anticipated to affect agricultural markets over the next few years. The “Organisation for Economic Cooperation and Development (OECD)” emphasizes how slower economic growth may have an influence on trade, GHG emissions, farm livelihoods, and food security. According to the report, the magnitude of these influences depends, among other things, on the sternness of the decline in global “gross domestic product (GDP)” [58].

Concerns over the safety of the world's food supply, particularly in developing nations, have increased as a result of CV-19's effects on the economy and agriculture [6, 59]. In addition to the limited research done on the macroimpacts of CV-19 on food security in specific countries, food security is an important factor that is impacted by global crises. In this regard, Rad et al. [6], in their study, attempt to examine the dynamic effects of CV-19 on food security in Iran as well as the country's economic and environmental problems. They conducted a survey with the hypothesis that CV-19 had no impact on Iran's food security. They used the systematic review approach to gather the data, including indices and statistics, from national databases, research papers, field observations, and interviews in order to address this fundamental hypothesis. According to preliminary findings from their study, CV-19 has a huge impact on Iran's economy, agriculture, and food security through a number of important mechanisms, which resulted in a 30% decline in the purchasing power parity in 2020 and a large increase in food costs compared to 2019. On the other hand, Iran's growing environmental restrictions decrease the agriculture sector's ability to play a significant role in the economy and guarantee food security. In this regard, CV-19 pushes the national budget and programs to confront the country's growing ecological restrictions.

The findings of a recent review study by Hassen and El Bilali [60] on the impacts of the CV-19 pandemic on food security and food consumption using the preliminary insights from the region of the Gulf Cooperation Council support the lack of data regarding the impact of the pandemic on diets and food-related behaviors in the region. In fact, the focus of the majority of academic studies on the effects of the CV-19 pandemic on food systems and diet has been on Western and Southern Europe, North America, and China [61]. In contrast, developing nations have generally received less attention, especially those in the neighborhood of the Gulf Cooperation Council. The CV-19 crisis has also highlighted the reality that, in terms of food security, nutrition security is more crucial than anything else. It might enable the Gulf States to combat food-related illnesses like obesity and diabetes with greater vigor. Policy actions might range from taxing foods high in carbohydrates and sugars and reporting requirements to school lunches and awareness programs [62].

As reported by Aaron et al. [63], while the self-reported livelihood impact of CV-19 was linked to a reduction in income, they also found that there was little variation in the correlation between the affordability of necessary items and the availability of food in families and markets in Vietnam. Self-determination of a significant economic impact may indicate a relative improvement in the household's prepandemic socioeconomic situation.

In order to prevent pandemic-caused food crises, Caballero-Anthony et al. [64] study how the CV-19 pandemic has affected food security in Asia and what steps nations might take to “pandemic-proof” their citizens' food security. It examines Singapore's methods for ensuring food security as prospective models for nations that both produce and import food. It also offers a plan for preventing and lessening the severe effects of pandemics on food security.

Also, in rural Sub-Saharan Africa, CV-19 has altered food consumption habits and hampered the food supply chain [59, 65, 66]. Senegal's production of four essential grains, including rice, maize, sorghum, and millet, was altered by restrictions on access to agricultural labor and inputs [67]. Middendorf et al. [68] assessed the pandemic's effects on Senegalese families' food security and way of life and found that 82.50% of households had trouble getting enough food. These studies showed how CV-19 could compromise the food supply chain in developing nations [69].  Figure 6 illustrates how CV-19 affects the food supply chain dynamically and demonstrates how rising food prices ultimately exacerbate poverty and food insecurity as adapted from Rad et al. [6].

Aside from the CV-19 pandemic's complex economic impacts, ecological limitations such as water deficiency, extreme soil erosion, salinity, deforestation, and natural adversities have critical consequences for global food security [70, 71]. As a result, CV-19 harms and disrupts the agriculture industry directly and indirectly by restricting the production of specific crops and disobeying environmental protection laws due to financial losses [72]. This is due to the potential threat that enduring ecological issues like soil erosion and salinity pose to future sustainable agricultural output [6, 73].

## 6. Conclusion, Recommendations, and Future Prospects

At the moment, the CV-19 issue is starting to take an erratic outline and it is alleged that most experts are likely to miss some aspects of the analysis. Although there are several reports that the CV-19 pandemic has instigated momentous adverse consequences, owing to the advancement in scientific researches, there is a possibility of relief since there is presently some positive information regarding the CV-19 virus vaccines.

However, from the meteorological perspective, the global response to the catastrophe ensuing from the CV-19 pandemic has a great influence on the reduction of GF, the reduction in the burning of fossil fuels from automobile and industrial devices, and the reduction in the other ensuing factors of GHGs emission such as CO_2_ and NO_2_ (which is one of the major drives for GW and climate change together with other environmental effluences during the CV-19 pandemic). Allegedly, these positive atmospheric environmental consequences are momentary. However, from all the reports on the influences of the CV-19 on the environment, it will not be far from the truth to conclude that there is a possible connection between the CV-19 pandemic and GHG emission.

The pertinent question is that, *since the CV-19 pandemic era experienced some level of environmental boosts, should we now crave for the pandemic to continue?* Of course, no. From the authors' respective personal viewpoints, all we have to do in sustaining these environmental boosts relished during the CV-19 pandemic era is the *green economy*. Consequently, to protect the environment, the combined effort of the countries should be domineering. It is therefore suggested that further advanced studies that would evolve the conduct of NanoTech and NanoBTech research to extenuating its impacts of GW regarding climate change and other environmental complications should be carried out. The positive influence of the CV-19 pandemic on the environment should be strengthened, to align and capitalize on the ensuing positive consequences of CV-19 for future prospects. Correspondingly, continuous prospects for impending researches and the provision for the scientific and theoretical course for the utilization of NanoTech and NanoBTech mechanisms for climate change studies should be strengthened. Therefore, appropriate approaches for longstanding benefits from the CV-19 pandemic together with sustainable atmospheric environmental management is necessary and should be rejuvenated.

Since it has been established that the CV-19's effects and ecological restrictions interact, support for small-scale farming and agricultural research initiatives may be halted due to the large financial loss. Governments must therefore promote ecofriendly legislation and sustainable agricultural practices to increase food security and environmental health. During a pandemic such as the CV-19 outbreak period, it is imperative to establish sustainable agriculture policies while taking ecological restrictions into account. Future research may therefore focus on developing agroecology training programs, accelerating agricultural projects through environmentally friendly methods, and supporting small-scale farming initiatives by offering site-specific solutions, automated tools, and novel breeds of seeds and plants to compensate for the long-term economic effects of the postpandemic on the agricultural sector.

The evolutions and developments in recent scientific outlooks such as NanoTech and NanoBTech tools for analyzing the climatic settings could have the possibility of combatting the effects of GW vis-à-vis climate change. Obviously, nanomaterials/bionanomaterials utilized in the nanotechnology and nanobiotechnology domains have demonstrated significant potential benefits in several environmental studies such as water technology and removal of heavy metals. Also, technological devices on the possibilities of using artificial intelligence (AI), big data, Internet of Things (IoT), and machine learning, particularly the affordable and ecofriendly ones (green computing) in the manipulation and tracking of the consumable energy and GHG emission, for developing analytical devices and more efficient ecosystem as well as reporting findings in accessible form should be enhanced.

## Figures and Tables

**Figure 1:** Summary of both the positive and negative environmental effects of CV-19 [26].

**Figure 2:** Influence of CV-19 on the various mechanisms of the ecosystem (water, soil, and air) [26].

**Figure 3:** Published articles in indexed journals as retrieved from the Scopus database employing the short statement “environmental impacts of CV-19” over the last year (from 2020 to 12 October, 2021).

**Figure 4:** GF volumes for the top 30 GasF nations between 2016 and 2020 [57].

**Figure 5:** GasF intensity for the topmost 30 GasF nations between 2016 and 2020 [57].

**Figure 6:** An illustration of how the CV-19's dynamic mechanisms threaten food security as adapted from Rad et al. [6].

**Table 1:** The emission sources of some of the utmost GHGs.

GHGs	Means of entering the atmosphere
CO_2_	BFFS from natural gas, petroleum resource, and coal. Solid waste, trees, and other biological resources. Also, as a consequence of certain chemical reactions such as GF, the manufacture of cement.

CH_4_	During the production and transportation of petroleum resources and coal. During most agricultural activities and from farm animals (livestock) and land use. During decaying activities of organic waste.

N_2_O	BFFS. During agricultural activities, industrial activities, remediation of wastewater, and land use. From solid waste.

Fluorinated gases such as CFCs, HCFC, and halon as well as synthesized SHF, HFC, nitrogen trifluoride, and perfluorocarbons	During various industrial activities.

## Data Availability

Completely, data produced or investigated during this work were involved in this submitted article.
